This article has been retracted.

# Automated Diagnosis and Localization of Melanoma from Skin Histopathology Slides Using Deep Learning: A Multicenter Study

**DOI:** 10.1155/2021/5972962

**Published:** 2021-10-26

**Authors:** Tao Li, Peizhen Xie, Jie Liu, Mingliang Chen, Shuang Zhao, Wenjie Kang, Ke Zuo, Fangfang Li

**Affiliations:** ^1^National University of Defense Technology, Changsha 410073, China; ^2^The Department of Dermatology, Xiangya Hospital, Central South University, Changsha 410008, China; ^3^Hunan Key Laboratory of Skin Cancer and Psoriasis, Changsha 410005, China; ^4^Hunan Engineering Research Center of Skin Health and Disease, Changsha 410005, China; ^5^Hunan Provincial Key Laboratory of Network Investigational Technology, Hunan Police Academy, Changsha 410138, China; ^6^Key Laboratory of Police Internet of Things Application Ministry of Public Security, Changsha 410138, China

## Abstract

In traditional hospital systems, diagnosis and localization of melanoma are the critical challenges for pathological analysis, treatment instructions, and prognosis evaluation particularly in skin diseases. In literature, various studies have been reported to address these issues; however, a prominent smart diagnosis system is needed to be developed for the smart healthcare system. In this study, a deep learning-enabled diagnostic system is proposed and implemented that it has the capacity to automatically detect malignant melanoma in whole slide images (WSIs). In this system, the convolutional neural network (CNN), sophisticated statistical method, and image processing algorithms were integrated and implemented to locate benign and malignant lesions which are extremely useful in the diagnoses process of melanoma disease. To verify the exceptional performance of the proposed scheme, it is implemented in a multicenter database, which has 701 WSIs (641 WSIs from Central South University Xiangya Hospital (CSUXH) and 60 WSIs from the Cancer Genome Atlas (TCGA)). Experimental results have verified that the proposed system has achieved an area under the receiver operating characteristic curve (AUROC) of 0.971. Furthermore, the lesion area on the WSIs is represented by its degree of malignancy. These results show that the proposed system has the capacity to fully automate the diagnosis and localization problem of the melanoma in the smart healthcare systems.

## 1. Introduction

According to the Global Cancer Statistics of 2018, approximately 120,000 patients with skin cancer succumb to the disease each year, while another 1,300,000 cases are diagnosed [1]. Melanoma skin cancer, which is assumed as the most server cancer type, causes nearly half of skin cancer deaths [2]. Thus, sophisticated and well-trained diagnosis methods are needed to be developed to minimize the death ratio. Currently, the most accurate and precise diagnosis method with maximum successful treatment ratio for melanoma cancer is the accurate diagnosis of hematoxylin and eosin- (H&E-) stained tissue slides [3]. However, this method is computationally expensive and time consuming. Therefore, it is urgent and critical to develop a fast, accurate, and high-precise method to assist pathologists in the diagnostic process of melanoma skin cancer.

Previous studies are on histopathology melanoma whole slide images (WSIs) have used computer-based image analysis approaches for cell segmentation and invasion depth prediction [4, 5]. These studies are based on topology, statistic, or machine learning approaches to predict expected ratio of the underlined skin cancer disease. However, due to the technological limitations, high performance of these studies is confined to the small handpicked dataset, which limits its clinical application. Therefore, an automated melanoma skin cancer prediction system is needed to be realized which is not only accurate and precise but at the same time generates fast results.

With the technological advances particularly in artificial intelligence-enabled diagnosis systems, deep learning-based approaches, specifically the convolutional neural network (CNN), have shown strong potential in the histopathology melanoma diagnosis process [6–11]. Achim Hekler et al. [12] have presented a deep learning method-enabled classification mechanism for the melanoma skin cancer which has obtained 81% accuracy on 695 slides (WSIs). Likewise, in the eyelid malignant melanoma identification task, the CNN and random forest-based smart diagnosis system have obtained areas under the receiver operating characteristic curve (AUROC) of 0.998 on 155 eyelids WSIs [13]. Kulkarni et al. have proposed a pathology-based computational method where the deep neural network was utilized for disease-specific survival prediction in early stage melanoma and has achieved an 0.905 AUROC [14]. However, these approaches are not well suited for the melanoma skin cancer disease prediction system which is capable to assist both pathologist and doctor in successful cure of the disease.

In this study, a deep learning-enabled smart and intelligent diagnosis system is proposed to automate both the identification and location processes of melanoma skin cancer disease in the hospitals. Main contributions to the research communication of this study are as follows.

- Development of a deep learning-enabled melanoma skin cancer disease prediction system with maximum possible ratio of the accuracy and precision metrics, respectively
- Develop and realize a multicenter melanoma database to speed up the diagnosis process with high accuracy ratio
- A deep learning-based diagnosis system to identify melanoma at the WSI-level
- Effective utilization of the heat maps to show the lesion area located on WSIs

The rest of the manuscript is organized as follows. In Section 2, the proposed methodology is described and presented in detail where the dataset, which is used during the experimental study of this study, is elaborated. In Section 3, the proposed work is described in detail, which is followed by the simulation section and discussion. Finally, concluding remarks and further perspective are provided.

## 2. Proposed Methodology

The deep learning-based WSI diagnostic framework was designed for skin tumor classification and location at various possible levels in the smart healthcare systems. The proposed system is divided into four different parts which is shown in Figure 1. The initial part, which is the preparation of patch, tiles WSI into patches and selects only those which are nonblank or having some values. Moreover, the proposed system has generated a patch-level classification by using the CNN in the second part as shown in Figure 1. The third part derives the WSI-level diagnosis using the WSI-level inference method. Finally, the proposed scheme is able to get the lesion area by generating the WSI-level visualization heat map in the fourth part as shown in Figure 1.

Patch preparation: four phases or part of the proposed scheme are as follows.

- WSIs: tiling WSIs into various possible patches
- Model inference: generating patch-level prediction using ResNet50 which is based on the CNN
- WSI diagnosis: deriving the WSI-level diagnosis using WSI-level inference information
- Lesion location: depict the location of the lesion area within image

### 2.1. Dataset

The proposed experimental study was performed under the Declaration of Helsinki Principles which has the capacity to build a multicenter database involving 701 H&E-stained whole-slide histopathology images from 583 patients in different hospitals [15]. Every WSI, which is used in the proposed study, was collected by cooperating with the Central South University Xiangya Hospital (CSUXH) and the Cancer Genome Atlas (TCGA). Experimental data were provided by these institutes where proper MOUs were signed. The relevant clinicopathological information is given in Table 1 with various metrics such as sex, age, and facility.

In the proposed deep learning-enabled smart diagnosis system, WSIs of four common skin diseases, which include melanoma, compound nevi, junctional nevi, and intradermal nevi, were contained in the dataset. However, the proposed system has selected those WSIs which are both dermis and epidermis. Furthermore, all WSIs are assumed to be clear enough to make the diagnosis process accurate and precise. Annotations of WSIs, outer margin of lesion areas, and normal areas were provided by pathologists to the proposed system.

For model training and testing, the dataset was randomly divided into training (70%), validation (15%), and test (15%) sets. Furthermore, the WSIs of one patient is only divided into one of the three sets that is training, validation, and testing. The source and disease distribution of WSIs in three sets are the same as that in the WSI dataset. The training and test sets were used for model training, and the validation set was used for the framework test. Moreover, images from the test and validation sets were blinded from the algorithm before the training process.

#### 2.1.1. Patch Preparation

Due to the enormous size of WSI (bigger than 100,000 × 100,000 pixels), the CNN model could not directly make inferences using raw WSIs. WSI was tiled into nonoverlapping 224 × 224 pixel patches for patch-level inference at a magnification of 20 × (0.5 *μ*m/pixel). In general, a WSI may contain 40–80% of white background. These patches with the background are significantly increasing the computational cost but with no diagnosis information. Therefore, the proposed system has used Otsu's method [16], which is a traditional method for image thresholding to filter all the irrelevant backgrounds while preserving the tissue patches for model inference.

#### 2.1.2. Patch-Level Inference with the CNN

WSI includes the lesions and a large amount of normal tissue (collagen and adipocyte) which are ranging from 10% to 50% of the WSI area in the proposed system. Moreover, these normal tissues are almost irrelevant to the diagnosis process. Therefore, a precise and accurate extraction of lesion features from the large WSIs is crucial to make the diagnosis process more effective and successful. In patch-level inference, a deep learning-based method was used to distinguish melanoma, intradermal nevi, junctional nevi, compound nevi, and normal tissue. Especially, a ResNet50 model was selected, which has minimum possible parameters, and its recognition capabilities are far beyond the expectations [17]. Furthermore, in the proposed model training process, we have used a cross-entropy loss and stochastic gradient descent (SGD) based optimization, particularly with a learning rate of 0.01, momentum of 0.9, and the weight decay of 0.0001. The model was trained in a single TITAN RTX GPU.

#### 2.1.3. WSI Inference Process

In order to classify the WSI-level interference processes, the counting method and averaging method were used. The counting and the averaging methods are classical statistical methods which are used for the classification of various tasks [18]. In the counting method, we have aggregated the WSI-level classification result by counting the percentage of patches in each disease class. Moreover, in the averaging method, the WSI-level classification result was aggregated by averaging the predicted scores of patches.

#### 2.1.4. Lesion Location

Lesion location shows the diagnostic basis of the proposed model to predict the expected results, which is critical for pathologists to understand why the model makes its decision. The lesion areas were located using the probability heat maps method, a data visualization technique that shows the magnitude of probability as color in two dimensions. Moreover, the probability heat map is obtained by feeding the malignancy probability back into the WSI. The lesion area of a specific class is marked in deep red, while other parts are not marked.

## 3. Experiment Results and Evaluations

To verify the expected performance of the proposed deep learning-enabled melanoma skin cancer disease prediction system, various experiments were performed on both benchmark datasets and real time datasets. The proposed scheme performance particularly in terms of the expected accuracy and precision ratio were evaluated and compared with the existing state of the art techniques in the smart healthcare systems.

### 3.1. The Framework Performs Effectively in Melanoma Classification

In order to validate and evaluate performance of the proposed deep learning-enabled classification system in the WSI-level melanoma classification task, we have used the counting and averaging methods to calculate various results. The receiver operating characteristic (ROC) curves are shown in Figure 2(a), which depicts performance of the proposed system in terms of sensitivity metrics. The averaging method (AUROC of 0.971) has achieved a slightly higher performance than the counting method (AUROC of 0.963), with a confidence interval (CI) of 0.952–0.990 and a *p* value of 0.039. Moreover, the precision-recall curves are shown in Figure 2(b). Area under the precision-recall curve (AUPRC) of the averaging method is 0.935. Furthermore, the AUPRC of the counting method is 0.926. The result shows that the averaging method is more suitable than the counting method in melanoma WSI diagnosis classification and prediction processes to assist phytologist in the diagnosis process.

### 3.2. Accuracy of the Proposed System to Locate the Lesion Area in WSI Levels

Generally, valuable lesion region to the pathologists occupies no more than 50% of the WSI. Therefore, the proposed system has provided additional lesion location information than the diagnosis results only which is very helpful or the pathologists particularly in the smart healthcare systems where maximum activities are needed to be automated. Furthermore, we have evaluated the lesion location ability of the proposed method in the test set dataset and compared it with existing approaches. The heat maps are shown in Figure 3. In the proposed deep learning-based method, the lesion area is visualized by the probabilistic heat map procedure and color shade is proportional to the classification probability. The outlines indicate the lesion area boundary, as shown in Figure 3.

## 4. Discussion

In this study, we have presented an automated WSI diagnostic system which is based on deep learning for melanoma diagnosis and lesion localization. For this purpose, we have generated a multicenter database which involves around 701 WSIs of 583 patients from CSUXH and TCGA. The proposed deep learning-based model provides an accurate and robust automated method for the melanoma diagnosis at the WSI level in the smart healthcare systems. Additionally, probabilistic heat maps are used to show the lesion areas, which could help experts locate the lesion areas quickly.

The deep learning and deep learning-enabled neural networks are notoriously data hungry; conclusively, more data and distinct features are needed to make the proposed system accurate and precise. For this purpose, effective features or data extraction methods are needed to be adopted in the proposed setup. Additionally, the size of the dataset and the diversity of samples are responsible for the reliability of deep learning-based studies. The WSI-level melanoma diagnostic model achieves a high diagnosis accuracy (AUROC of the averaging method: 0.971; AUROC of the counting method: 0.963). Nevertheless, authors have augured that their model's reliability was questionable because of the overlap in patients between train, validation, and test sets due to the lack of data. In this study, a multicenter dataset containing 701 WSIs for developing of the proposed system was utilized which was generated with cooperation of the two well-known hospitals as described above. The dataset contains WSIs of different ages, genders, and organs, and several metastatic melanoma slides were collected to increase melanoma morphology diversity.

The proposed framework has achieved comparable accuracy and precision in WSI-level melanoma diagnosis on a multicenter multiracial database which is an indication of how strong generalization ability of the proposed approach is? Meanwhile, the proposed deep learning-enabled method provides pathologists with additional diagnosis information, the lesion location. As shown in Figure 3, the area of higher malignant probability overlaps with the core lesion area. Although the lesion location cannot fully indicate the lesion area, additional diagnostic or evaluation of information is helpful for the pathologists to understand the diagnostic basis of the model. Last, the proposed model is the best possible assist software, which is designed specifically for the pathologists in potential lesion discovery.

Conclusively, we have proposed a deep learning-based pathology diagnosis system for melanoma WSI classification and generated a multicenter WSI database for model training and testing purposes. The proposed model has the capacity to provide a fully automatic approach for the classification of melanoma and lesion location, which could assist the pathological diagnosis of melanoma diseases.

## 5. Conclusion and Future Work

In this study, a deep learning-enabled diagnostic system was proposed and implemented that has the capacity to automatically detect malignant melanoma in whole slide images (WSIs). In the proposed system, the convolutional neural network (CNN), sophisticated statistical method, and image processing algorithms were integrated and implemented to locate benign and malignant lesions which are extremely useful in the diagnoses process of melanoma disease. To verify the exceptional performance of the proposed scheme, it was implemented in a multicenter database, which has 701 WSIs (641 WSIs from Central South University Xiangya Hospital (CSUXH) and 60 WSIs from the Cancer Genome Atlas (TCGA). Experimental results have been verified that the proposed system has achieved an area under the receiver operating characteristic curve (AUROC) of 0.971. Furthermore, the lesion area on WSIs were represented by its degree of malignancy. These results show that the proposed system has the capacity to fully automate the diagnosis and localization problem of the melanoma in the smart healthcare systems.

In future, we are eager to enhance the operational capabilities of the proposed models particularly in terms of various other cancer diseases in general and skin cancer in particular.

## Figures and Tables

**Figure 1:** The deep learning-based WSI diagnostic framework.

**Figure 2:** Performance comparison of the counting method and averaging method. (a) ROC of counting and averaging methods in the WSI-level melanoma classification task is represented, respectively. (b) PRC of both counting and averaging methods in the WSI-level melanoma classification task.

**Figure 3:** Lesion location. The red line outlines the ground truth labelled by the pathologist and the heat map, with the blue line showing the lesion area located by the model. (a). Lesion location in melanoma WSI. (b). Lesion location in compound nevi WSI. (c). Lesion location in intradermal nevi WSI. (d). Lesion location in junctional nevi WSI.

**Table 1:** Characteristics of the database.

		MM		IN		CN		JN	
		*n*	%	*n*	%	*n*	%	*n*	%
Sex	Male	114	45.2	45	23.9	39	32.8	45	31.7
	Female	138	54.8	143	76.1	80	67.2	97	68.3

Age	Mean	55.5	—	29.7	—	19.8	—	31	—
	SD	14.0	—	11.6	—	10.4	—	13.1	—

Facility	CSUXH	192	76.2	188	100.0	119	100.0	142	100.0
	TCGA	60	23.8	—	—	—	—	—	—

MM, melanoma; IN, intradermal nevi; CN, compound nevi; JN, junctional nevi; SD, standard deviation; CSUXH, Central South University Xiangya Hospital; TCGA, The Cancer Genome Atlas.

## Data Availability

The data of CSUXH used and/or analyzed during the current study are available from the corresponding author upon request. The data of TCGA are available from https://portal.gdc.cancer.gov/.

## References

[1] Stewart B., Wild C. (2019). *World Cancer Report 2014*.

[2] Schadendorf D., van Akkooi A. C. J., Berking C. (2018). Melanoma. *The Lancet*.

[3] https://pubmed.ncbi.nlm.nih.gov/26389482/.

[4] Lu C., Mahmood M., Jha N., Mandal M. (2013). Automated segmentation of the melanocytes in skin histopathological images. *IEEE Journal of Biomedical and Health Informatics*.

[5] Xu H., Berendt R., Jha N., Mandal M. (2017). Automatic measurement of melanoma depth of invasion in skin histopathological images. *Micron*.

[6] LeCun Y., Bengio Y., Hinton G. (2015). Deep learning. *Nature*.

[7] Liang H., Tsui B. Y., Ni H. (2019). Evaluation and accurate diagnoses of pediatric diseases using artificial intelligence. *Nature Medicine*.

[8] Zhang Z., Chen P., McGough M. (2019). Pathologist-level interpretable whole-slide cancer diagnosis with deep learning. *Nature Machine Intelligence*.

[9] Kather J. N., Krisam J., Charoentong P. (2019). Predicting survival from colorectal cancer histology slides using deep learning: a retrospective multicenter study. *PLoS Medicine*.

[10] Zeng C., Nan Y., Xu F. (2020). Identification of glomerular lesions and intrinsic glomerular cell types in kidney diseases via deep learning. *The Journal of Pathology*.

[11] Campanella G., Hanna M. G., Geneslaw L. (2019). Clinical-grade computational pathology using weakly supervised deep learning on whole slide images. *Nature Medicine*.

[12] Hekler A., Utikal J. S., Enk A. H. (2019). Pathologist-level classification of histopathological melanoma images with deep neural networks. *European Journal of Cancer*.

[13] Wang L., Ding L., Liu Z. (2020). Automated identification of malignancy in whole-slide pathological images: identification of eyelid malignant melanoma in gigapixel pathological slides using deep learning. *British Journal of Ophthalmology*.

[14] Kulkarni P. M., Robinson E. J., Sarin Pradhan J. (2020). Deep learning based on standard H&E images of primary melanoma tumors identifies patients at risk for visceral recurrence and death. *Clinical Cancer Research*.

[15] Association GAotW (2014). World medical association declaration of Helsinki: ethical principles for medical research involving human subjects. *Journal of the American College of Dentists*.

[16] Otsu N. (1979). A threshold selection method from gray-level histograms. *IEEE transactions on systems, man, and cybernetics*.

[17] He K., Zhang X., Ren S., Sun J. Deep residual learning for image recognition.

[18] Coudray N., Ocampo P. S., Sakellaropoulos T. (2018). Classification and mutation prediction from non-small cell lung cancer histopathology images using deep learning. *Nature Medicine*.

